# Combining Rhythm Information between Heartbeats and BiLSTM-Treg Algorithm for Intelligent Beat Classification of Arrhythmia

**DOI:** 10.1155/2021/8642576

**Published:** 2021-12-13

**Authors:** Jinliang Yao, Runchuan Li, Shengya Shen, Wenzhi Zhang, Yan Peng, Gang Chen, Zongmin Wang

**Affiliations:** ^1^School of Information Engineering, Zhengzhou University, Zhengzhou 450000, China; ^2^Collaborative Innovation Center for Internet Healthcare, Zhengzhou University, Zhengzhou 450000, China; ^3^Zhengzhou College of Economics and Business, Zhengzhou, Henan 450000, China

## Abstract

Arrhythmia is a cardiovascular disease that seriously affects human health. The identification and diagnosis of arrhythmia is an effective means of preventing most heart diseases. In this paper, a BiLSTM-Treg algorithm that integrates rhythm information is proposed to realize the automatic classification of arrhythmia. Firstly, the discrete wavelet transform is used to denoise the ECG signal, based on which we performed heartbeat segmentation and preserved the timing relationship between heartbeats. Then, different heartbeat segment lengths and the BiLSTM network model are used to conduct multiple experiments to select the optimal heartbeat segment length. Finally, the tree regularization method is used to optimize the BiLSTM network model to improve classification accuracy. And the interpretability of the neural network model is analyzed by analyzing the simulated decision tree generated in the tree regularization method. This method divides the heartbeat into five categories (nonectopic (N), supraventricular ectopic (S), ventricular ectopic (V), fused heartbeats (F), and unknown heartbeats (Q)) and is validated on the MIT-BIH arrhythmia database. The results show that the overall classification accuracy of the algorithm is 99.32%. Compared with other methods of classifying heartbeat, the BiLSTM-Treg network model algorithm proposed in this paper not only improves the classification accuracy and obtains higher sensitivity and positive predictive value but also has higher interpretability.

## 1. Introduction

With the improvement of people's living standards, the incidence and mortality of cardiovascular diseases are increasing year by year and are accompanied by a younger trend [1]. Arrhythmia is a common cardiovascular disease, which may endanger people's lives in serious cases [2]. Therefore, the accurate detection of arrhythmia to prevent heart disease has a very important significance. Electrocardiogram (ECG), as a comprehensive expression of cardiac electrical activity on the body surface, contains a wealth of physiological and pathological information reflecting cardiac rhythm and electrical conduction and is one of the important bases for diagnosis of heart disease and evaluation of cardiac function [3]. Different types of arrhythmias can be identified and diagnosed by analyzing the ECG waveform. Traditional ECG waveform analysis is performed manually by medical personnel, who need to give a diagnosis based on cardiovascular disease diagnosis rules and personal experience. Due to the individual differences of patients and the complexity of diseases, there are many types of ECG. In addition, some arrhythmias occur only occasionally in the daily life of the patients, and the ECG data need to be recorded for a long time. Therefore, the amount of collected ECG data is huge, which brings a heavy burden to doctors. Under the circumstances, mistakes, missed inspections, or misdetections easily occur. With the rapid development of computer technology and electronic information technology, the computer has become an indispensable and important tool of medical modernization, and computer-aided medical treatment has penetrated into every corner of medical service [4]. In recent years, increasing attention has been paid to the study of computer-aided analysis algorithms for electrocardiography, particularly those that can accurately and rapidly identify and diagnose arrhythmias. The automatic classification and diagnosis algorithm of ECG signals can save doctors' time by helping them better judge the symptoms of arrhythmia quickly. In addition, it can provide good healthcare in areas where medical resources are scarce.

This paper presents a beat classification method based on the time-series network, which integrates the interheartbeat rhythm information. This method is based on tree regularization constraints and the BiLSTM neural network model. This method improves the accuracy of heartbeat classification. And the interpretability of the proposed algorithm is analyzed by tree regularization constraints and feature analysis. The main contributions of this work are as follows:

1. A time-series BiLSTM-Treg algorithm was designed to classify the beats, which combined the information of the beats so that the deep neural network could learn more rhythm information between heartbeats.
2. A tree regularization method for the heartbeat classification model is proposed to optimize the BiLSTM-Treg algorithm and improve the generalization ability of the neural network model.
3. By analyzing the key nodes of the simulated decision tree in tree regularization, the concerns in the learning process of the BiLSTM-Treg algorithm are analyzed, and the interpretability of the model is analyzed to a certain extent.
4. Compared with other deep learning methods, the proposed BiLSTM-Treg algorithm improves the accuracy of heartbeat classification and reduces doctor's misdiagnosis rate to a certain extent

## 2. Related Work

The diagnosis of early arrhythmia is mainly the doctor's manual analysis of ECG waveform, which requires the doctor to have a professional medical theoretical basis and rich clinical experience. Because of the diversity of arrhythmia and the complexity of the ECG waveform, this method cannot meet the needs of patients. With the development of artificial intelligence, the classification of arrhythmia using intelligent processing technology has become a hot topic in recent years.

In the 1950s, the automatic analysis technology of ECG signals has appeared in the field of ECG research. At first, only ECG filtering processing technology developed relatively mature. Later, with the continuous development of technology, automatic detection and diagnosis of arrhythmia disease also began to be continuously explored by researchers. In the past decades, domestic and foreign ECG researchers have proposed a variety of heartbeat classification methods. These methods can be divided into two categories from the perspective of whether manual feature extraction of ECG signals is needed: feature engineering-based classification methods and deep learning-based methods [5]. Traditional rule-based and machine-learning-based heartbeat classification methods both require manual feature extraction.

### 2.1. Heartbeat Classification Method Based on Feature Engineering

Feature engineering is to process a series of original data and extract the features as the input of the model to improve the performance of the model. Feature engineering mainly includes three aspects: feature selection, feature extraction, and feature construction. Feature extraction is the key step of ECG signal classification and recognition, and the extracted feature quality will affect the accuracy of ECG signal classification and recognition [6]. Generally, the features of ECG signals extracted by researchers mainly include morphological features [7], interphase features [8, 9], wavelet transform features [10], higher-order statistics (HOS) [9, 11], Hermite basis function (HBF) [12], QRS amplitude vector [13], and QRS composite wave area [14]. Then machine-learning algorithms are used for classification, such as the KNN algorithm [15], support vector machine (SVM) [7], and random forest [9]. Zhu et al. [7] extracted the ECG morphological features and used the SVM algorithm to classify the heartbeat, achieving a high classification accuracy. Yang et al. [9] extracted a variety of features, including RR interval, wavelet coefficient, and high-order statistics, and then used the random forest classifier based on an extreme learning machine to detect arrhythmias. Ji et al. [15] proposed a multifeature combination and stacked DWKNN algorithm to classify arrhythmias. The effects of different characteristic combinations on the classification of the heartbeat were analyzed.

Although this method based on feature engineering can also achieve relatively high classification accuracy, because of the complex waveform and poor anti-interference ability of ECG signal, the features extracted by hand often produce the human error. And the features of the manual design are very dependent on the prior knowledge of the researcher. Deep learning has the advantage of automatically extracting features and classification, which well solves a series of problems caused by manual feature extraction.

### 2.2. Heartbeat Classification Method Based on Deep Learning

The deep learning model has become a common model for ECG data classification [16]. Compared with the feature engineering-based ECG classification method, the deep learning method, which uses original data rather than manually extracted features as input, can achieve better classification performance. In the deep learning method, researchers use the nonlinear transformation of hidden layers in the network to automatically obtain effective features and transform the original features into different new feature spaces by changing the structure of hidden layers in the network and the way of stacking [17], so as to make full use of the rich hidden information in the data and improve the classification accuracy.

Recently, some researchers [18, 19] have used a deep neural network model for automatic classification of ECG signals. Ji et al. [20] proposed an ECG classification system based on Faster R-CNN. One-dimensional ECG signal is converted into two-dimensional image as the input of neural network to realize the classification of arrhythmias. Akarya et al. [21] proposed a 9-layer deep convolutional neural network (CNN) for automatic recognition of ECG signals. The original ECG signal and the ECG signal filtered out the high-frequency noise were used to classify the heartbeat, and the accuracy rates were 94.03% and 93.47%, respectively. Khan et al. [22] used the long short-term memory network (LSTM) to automatically identify 16 different types of arrhythmias. Wu et al. [23] proposed a heartbeat classification algorithm that integrated CNN and BiLSTM deep learning models and extracted the morphological and temporal features of heartbeat, respectively, by using CNN and BiLSTM. Li et al. [24] proposed a BiLSTM-Attention Network model to distinguish different types of arrhythmias. Pandey et al. [25] applied the extracted features of wavelet, RR interval, morphology, and high-order statistics to BiLSTM to achieve the automatic classification of the heartbeat. Yildirim et al. [26] proposed a heartbeat classification model based on wavelet transform and BiLSTM network, which used wavelet to decompose ECG signals into signals of different frequency scales and used the signals as the input sequence of the BiLSTM model.

The classification method of ECG signals based on deep learning realizes the “end-to-end” learning mode, eliminates the manual design process of features, saves manpower, and makes the process of ECG classification simpler and more efficient. Although all the above studies cleverly used the deep neural network to classify ECG signals, the rhythm information between heartbeats has not been fully considered, the interpretability of the network has not been analyzed, and the classification accuracy needs to be improved.

## 3. Method

The heartbeat classification method of the BiLSTM-Treg algorithm that integrates rhythm information between heartbeats proposed in this paper mainly includes the following steps: firstly, the data are preprocessed to filter out the noise in the ECG signal and segment ECG signal into heartbeats. Secondly, the continuous single heartbeat is combined into heartbeat segments so that the rhythm information between the heartbeats can be retained. Then, the BiLSTM-Treg model was constructed and optimized. Finally, the heartbeats were classified.  Section 3.1 is the preprocessing part, Section 3.2 is the representation of the rhythm information part, and Section 3.3 is the model building and optimization part.

### 3.1. ECG Signal Preprocessing

The preprocessing stage is mainly denoising and segmentation of ECG signals. Generally speaking, the collected ECG signals inevitably contain noise due to the influence of equipment and human body itself [27], which mainly includes baseline drift, power frequency interference, and EMG interference. It is important to remove as much noise as possible from ECG signals before classifying them. Wavelet transform is a generalization of short-time Fourier transform (STFT) [28], which can perform time-frequency analysis of ECG signals well. Compared with the equally spaced time-frequency localization of STFT, wavelet transform can provide higher frequency resolution at low frequency and higher time resolution at high frequency. In this paper, discrete wavelet transform is used to denoise ECG signals, which can avoid losing important physiological details in ECG signals and better retain the characteristics of ECG signals. Because of the high regularity of the Daubechies wavelet, the reconstructed signal is relatively smooth. And the strength spectrum of the DB6 wavelet [29, 30] is focused on low frequencies. Its moderate filter length and moderate coefficient values, compared with the other wavelets, provide more smoothing and less shift in the ECG fiducials. Therefore, in order to obtain a good classification accuracy, this paper uses the DB6 wavelet in the Daubechies wavelet base to process ECG signals. In terms of implementation, we use python's open-source wavelet transform tool pywt. The discrete wavelet transform formula [31] is shown in (1) and (2).

(1) $$\begin{array}{c} W_{\Psi }\left(j,k\right)=\sum_{x}f\left(x\right)\Psi_{j,k}\left(x\right), \end{array}$$

(2) $$\begin{array}{c} \Psi_{j,k}\left(x\right)=a_{0}^{-J/2}\Psi \left(a_{0}^{-j}x-kb_{0}\right), \end{array}$$

where *W*_Ψ_(*j*, *k*) is the wavelet coefficient, Ψ_*j*,*k*_(*x*) is the discrete wavelet function at different scales and locations, *f*(*x*) is the input ECG signal, Ψ(*k*) is the wavelet basis function, and *j* is the order of the scale. The larger *j* is, the smaller the scale is, which means the higher the frequency is and the closer it is to the details. *k* is the offset of position. *a*_0_ is the scale parameter and *b*_0_ is the position parameter. Signal comparison before and after pretreatment with discrete wavelet transform is shown in Figure 1 and Figure 2.

Heartbeat segmentation is to divide an ECG record with a complete heartbeat as a unit [32]. A complete heartbeat should contain P wave, QRS compound wave, and *T* wave [33], as shown in Figure3(a). In this paper, the peak value of the *R* wave marked in the MIT-BIH database was used as the reference point for heartbeat segmentation, and 0.25s and 0.4s were extracted before and after the peak of *R*, as shown in Figure 3(b). We take this 0.65S data as a sample of a single heartbeat. For MIT-BIH ECG data with a sampling rate of 360HZ, we extracted 90 points before *R* peak and 144 points after *R* peak. Therefore, the reconstructed sample is 235 points.

### 3.2. Rhythm Information between Heartbeats

The rhythm information between heartbeats contained in the ECG is an important basis for doctors to diagnose heart diseases. Changes in ECG rhythm can reflect problems in different parts of the heart, which can help medical staff design more rational treatment plans. Common rhythm types are bigeminy, trigeminy, ventricular tachycardia, and atrial tachycardia.

*Bigeminy*. Every normal heartbeat is followed by a premature beat. And the occurrence of three or more groups in a row is called bigeminy. According to the type of premature beat, it can be divided into ventricular bigeminy and atrial bigeminy. For example, the rhythm change of N–V–N–V–N–V is ventricular bigeminy, and the rhythm change of N–S–N–S–N–S is atrial bigeminy.

*Trigeminy*. A premature beat occurs after every two normal heartbeats. And the occurrence of three or more groups in a row is called trigeminy. According to the type of premature beat, it can be divided into ventricular trigeminy and atrial trigeminy. For example, the rhythm change of N–N–V–N–N–V–N–N–V is ventricular trigeminy, and the rhythm change of N–N–S–N–N–S–N–N–S is atrial trigeminy. The ECG signal with ventricular trigeminy is shown in Figure 4.

*Ventricular Tachycardia*. Three or more consecutive ventricular premature beats are called ventricular tachycardia, such as the rhythm change V–V–V.

*Atrial Tachycardia*. Three or more consecutive atrial premature beats are called atrial tachycardia, such as the rhythm change S–S–S.

In addition, the appearance of certain types of heartbeats also reflects changes in ECG rhythm. For example, after a continuous ventricular tachycardia, a ventricular fusion heartbeat is often generated due to electrical signals from the sinus node, followed by ventricular capture. Therefore, ventricular fusion heartbeat and ventricular capture are important characteristics of ventricular tachycardia.

In this paper, this rhythmic information, which is beneficial to the classification of heartbeats, was integrated into the model. Specifically, in processing the dataset, successive single beats were grouped into segments, which preserved information about rhythm between beats. Then, the ECG data is input into the neural network model in the unit of heartbeat segment, which enables the model to make full use of the rhythm information contained in the heartbeat segment when identifying the heartbeat type and improves the classification accuracy. The length of the heartbeat segment is one of the key points of our study.

### 3.3. BiLSTM-Treg Algorithm

Recurrent neural network (RNN) is a kind of neural network with short-term memory ability, which is very effective in processing data with sequence characteristics. However, in deep neural networks, the gradient is unstable. The gradient close to the input layer is calculated based on the product of the gradients of the subsequent layers [34]. When the neural network has too many hidden layers or the input sequence of the RNN network is too long, it will cause the gradient near the input layer to vanish or blow up, which affects the performance of RNN to some extent. In order to solve this problem, Hochreiter et al. [35] proposed the long short-term memory network (LSTM) in 1997. By adding gating units into RNN, the network can choose whether to retain the historical information so as to solve the problem of gradient disappearance and gradient explosion caused by long-term dependence of the RNN network.

#### 3.3.1. BiLSTM Neural Network Structure

Compared with RNN, LSTM adds three gating units, which are input gate, forgetting gate, and output gate. In addition, there are two important parts of LSTM, namely, memory unit, and hidden state. The forgetting gate controls whether the information in the memory unit is discarded, the input gate controls whether the information of the current signal and hidden state is added to the memory unit, and the output gate determines the information output in the memory unit.  Figure 5 shows the unit structure of the LSTM, where *f*_*t*_, *i*_*t*_, and *o*_*t*_, respectively, represent the forgetting gate at the current moment, the input gate, and the output gate; *C*_*t*−1_ and *C*_*t*_, respectively, represent the state value of the memory unit at the previous moment and the current moment; *h*_*t*−1_ and *h*_*t*_, respectively, represent the hidden state at the previous moment and the current moment. *x*_*t*_ represents the input at the current moment, and ${\tilde{C}}_{t}$ is the candidate value of the memory unit at the current moment. *σ* and tanh represent the sigmoid activation function and tanh activation function, respectively.

The calculation process of LSTM can be expressed as equations (3–8):

(3) $$\begin{array}{c} i_{t}=sigmoi\;d\left(W_{i}x_{t}+U_{i}h_{t-1}+b_{i}\right), \end{array}$$

(4) $$\begin{array}{c} f_{t}=sigmoi\;d\left(W_{f}x_{t}+U_{f}h_{t-1}+b_{f}\right), \end{array}$$

(5) $$\begin{array}{c} o_{t}=sigmoi\;d\left(W_{o}x_{t}+U_{o}h_{t-1}+b_{o}\right), \end{array}$$

(6) $$\begin{array}{c} {\tilde{C}}_{t}=\tanh\left(W_{c}x_{t}+U_{c}h_{t-1}+b_{c}\right), \end{array}$$

(7) $$\begin{array}{c} C_{t}=f_{t}⊗C_{t-1}+i_{t}⊗{\tilde{C}}_{t}, \end{array}$$

(8) $$\begin{array}{c} y_{t}=h_{t}=o_{t}⊗\;\tanh\left(C_{t}\right). \end{array}$$

Formulas (3)–(6), respectively, represent the calculation formulas for the input gate *i*_*t*_, forget gate *f*_*t*_, output gate *o*_*t*_, and candidate value ${\tilde{C}}_{t}$ of the memory unit. They are all determined by the input data *x*_*t*_ at the current moment, the hidden state *h*_*t*−1_ at the previous moment, and their corresponding weight matrix, where *W*_*i*_, *W*_*f*_, *W*_*o*_, and *W*_*c*_ are the weight matrix of the current input *x*_*t*_; *U*_*i*_, *U*_*f*_, *U*_*o*_, and *U*_*c*_ represent the weight matrix of the hidden state *h*_*t*−1_ at the last moment; *b*_*i*_, *b*_*f*_, *b*_*o*_, and *b*_*c*_ are the corresponding bias items, respectively. These weight matrices and bias terms are trained by the way of gradient descent. Formula (7) indicates that the current moment memory unit *C*_*t*_ is adjusted by the current candidate unit ${\tilde{C}}_{t}$ and its own state *C*_*t*−1_ as well as the input gate and the forgetting gate. Finally, formula (8) indicates that the output at the current moment, that is, the hidden state at the current moment, is determined by the current memory unit *C*_*t*_ and the output gate.

One disadvantage of LSTM is that it cannot encode information upfront and can only use its past context, not its future context. In the classification of heartbeat, if the relevant information of the former and the latter can be obtained at the same time during the classification of the current heartbeat, the rhythm information of the heartbeat will be grasped more accurately, thus improving the classification accuracy of the current heartbeat. And BiLSTM solves this problem well [36]. In each BiLSTM layer, there are two independent LSTM to process sequences in two directions, respectively. The specific formula is shown in (9)–(11). At the time *t*, the hidden layer state *H*_*t*_ of BiLSTM obtains the heartbeat information $\overset{⟶}{h_{t}}$ before the time *t* through the forward LSTM and the heartbeat information $\overset{⟵}{h_{t}}$ after the time *t* through the backward LSTM and then carries out the weighted sum of $\overset{⟶}{h_{t}}$ and $\overset{⟵}{h_{t}}$, where $\overset{⟶}{W_{t}}$ and $\overset{\leftarrow }{W_{t}}$ are the corresponding weight matrices and *b*_*t*_ is the bias term.

(9) $$\begin{array}{c} \overset{⟶}{h_{t}}=\text{LSTM}\left(x_{t},\overset{⟶}{h_{t-1}}\right), \end{array}$$

(10) $$\begin{array}{c} \overset{⟵}{h_{t}}=\text{LSTM}\left(x_{t},\overset{⟵}{h_{t-1}}\right), \end{array}$$

(11) $$\begin{array}{c} H_{t}=\overset{⟶}{W_{t}}\overset{⟶}{h_{t}}+\overset{⟵}{W_{t}}\overset{⟵}{h_{t}}+b_{t}. \end{array}$$

#### 3.3.2. BiLSTM Network Based on Tree Regularization

In machine learning, there are many strategies designed to reduce model generalization errors, which are collectively referred to as regularization. The form of regularization is very simple, which is to add an additional term after the objective function to affect the selection of the optimal point of the objective function. The common regularization methods are L1 regularization and L2 regularization. The common regularization methods are L1 regularization and L2 regularization. The objective function is shown in equation (12), where *λ*Ψ(*W*) is a regular term.

(12) $$\begin{array}{c} \underset{W}{\min}\sum_{n=1}^{N}loss\left(y_{n},\hat{y_{n}}\left(x_{n},W\right)\right)+\lambda \Psi \left(W\right). \end{array}$$

Tree regularization is a new regularization method proposed by Wu et al. [37], which can not only effectively improve the generalization ability of the model but also analyze the interpretability of the model. The tree regularization method of deep network model interpretability is a postinterpretable method, that is, the method of applying model analysis after model training to make the model interpretable. This method looks for the decision tree representation of the deep network model and realizes the human understanding of the prediction results of the network model by improving the human simulability of the network model. The implementation method of tree regularization includes the following two stages. First, we train deep neural network while being closely modeled by decision trees. In this way, this decision tree can accurately simulate the prediction process of the network. Secondly, the complexity metric of the decision tree, the average path length (APL), is taken as the penalty term for model optimization. In this way, the neural network can be encouraged to generate simple decision trees and restricted to generate complex decision trees, which further makes the generated decision trees easier to be simulated by human beings. The decision tree generation formula can be expressed by (13) and (14), where *x*_*n*_ is the sample feature of the training set, $\hat{y_{n}}\left(x_{n},W\right)$ is the prediction label of the depth model, *W* is the weight matrix of the depth model, and $\hat{y_{tn}}$ is the prediction label of the decision tree. The reason why $\hat{y_{n}}$ is used as the input of the decision tree is to make $\hat{y_{tn}}$ and $\hat{y_{n}}$ as similar as possible so as to realize the purpose of using the decision tree to simulate the deep network.

(13) $$\begin{array}{c} \text{Tree}=Tra\mathrm{int}ree\left(\left\{x_{n},\hat{y_{n}}\left(x_{n},W\right)\right\}\right), \end{array}$$

(14) $$\begin{array}{c} \hat{y_{tn}}=Tree.pre\;di\;ct\left(x_{n}\right). \end{array}$$

The calculation formula of tree regularization is shown in (15), where Path *Length*(tree, *x*_*n*_) is the path length of the *n* sample and Ω(*W*) is the average path length, namely, the penalty term.

(15) $$\begin{array}{c} \Omega \left(W\right)=\frac{1}{N}\sum_{n}Path\;Length\left(tree,x_{n}\right). \end{array}$$

It can be seen from equation (15) that is not differentiable for network parameter *W*. Therefore, in order to use the gradient descent strategy in the network optimization process, Wu et al. [37] proposed the surrogate regularization function $\tilde{\Omega }\left(W\right)$, which can surrogate the previous APL calculation method, as shown in equations (16) and (17). By training a Multilayer Perceptron (MLP), the mapping relationship between the parameter vector W of the neural network model and APL is established. With W and APL as inputs to MLP, the objective function of MLP is shown in equation (17), where *ξ* represents the weight matrix of the MLP model, *ε* represents the regularization intensity, {*W*_*j*_, Ω(*W*_*j*_)} represents the known parameter vectors and their corresponding real APL datasets, and *J* represents the total number of datasets. Therefore, after using the surrogate model, the objective function of the BiLSTM network is shown in equation (18).

(16) $$\begin{array}{c} \tilde{\Omega }\left(W\right)\approx \frac{1}{N}\sum_{n}Path\;Length\left(tree,x_{n}\right), \end{array}$$

(17) $$\begin{array}{c} \underset{\xi }{\min}\sum_{j=1}^{J}{\left(\Omega \left(W_{j}\right)-\tilde{\Omega }\left(W_{j},\xi \right)\right)}^{2}+\varepsilon {\left\|\xi \right\|}_{2}^{2}, \end{array}$$

(18) $$\begin{array}{c} \underset{W}{\min}\sum_{n=1}^{N}loss\left(y_{n},\hat{y_{n}}\left(x_{n},W\right)\right)+\lambda \tilde{\Omega }\left(W\right). \end{array}$$

In this paper, tree regularization is used in the BiLSTM model to optimize the model, reduce the generalization error of the model, and improve the classification accuracy. At the same time, the generated simulated decision tree is used to analyze and understand how the BiLSTM model carries out heartbeat classification. The BiLSTM model using tree regularization is shown in Figure 6. Specifically, *x*_*t*_=[*x*_*t*1_, *x*_*t*2_,…, *x*_*t*235_, ] is used to represent a single heartbeat sample. The heartbeat segment composed of consecutive single heartbeats is used as the input of the network, and the number of single heartbeats in the heartbeat segment *t* is the timestep of the network. The model first uses BiLSTM to classify heartbeat. Secondly, the decision tree is used to simulate BiLSTM, and APL is calculated. Then, the MLP model is trained to get the surrogate regularization function $\tilde{\Omega }\left(W\right)$, and then $\tilde{\Omega }\left(W\right)$ is added to the objective function of the BiLSTM model for the next round of training.  Algoithm 1 describes the BiLSTM-Treg model algorithm.

## 4. Experiment

The processing and analysis of ECG signal is very important to the classification of the heartbeat. The research focus of this paper is on the construction and optimization of the model integrating rhythm information. According to the ANSI/AAMI EC57:2012 classification proposed by the Association for the Advancement of Medical Instruments (AAMI), arrhythmia can be divided into five categories: N (normal or bundle branch block), S (supraventricular ectopic beat), V (ventricular ectopic beat), F (fusion beat), and *Q* (beat not specified). On the basis of extracting continuous heartbeat segments, this experiment constructs a time-series network that integrates rhythm information between heartbeats and divides heartbeats into the above five types.

### 4.1. Experimental Environment

The model proposed in this paper is trained and tested on a PC workstation with Xeon(R)Silver-4114CPU, 32 GB memory, and Geforce2080Ti graphics card. The PC workstation runs on Ubuntu 18.04 system. And the algorithm is run under the TensorFlow-GPU V2.2.0 framework.

### 4.2. Experimental Data

A unified and authoritative standard database is the basis of the automatic analysis of ECG signals. In the research field of ECG signals, the MIT-BIH arrhythmia database is the most widely used database by researchers [38]. The database contains 48 records, each of which is about 30 minutes long, with about 650,000 sampling points and a sampling frequency of 360 Hz. Fifteen categories were labeled in the MIT-BIH arrhythmia database.  Table 1 is the corresponding table of the two heartbeat classification methods.

In this paper, we classified 109,454 heartbeats from the MIT-BIH arrhythmia database, including 90,595 N-type heartbeats; 2,781 heartbeats in the S category; 7,235 V-type heartbeats. The number of heartbeats in category F was only 802 and in *Q* was 8041. In this paper, 90% of the heartbeat data were randomly selected from the dataset as the training set and the remaining 10% as the test set. And the specific distribution of data is shown in Table 2.

### 4.3. Evaluation Metrics

In order to calculate the performance of the model for heartbeat classification, the classification results were divided into four categories: TP, FP, TN, and FN. Take N-type as an example; formulas (19)–(22), respectively, represent the calculation methods of type N true positive heartbeat (TP_N_), type N false-positive heartbeat (FP_N_), type N true negative heartbeat (TN_N_), and type N false-negative heartbeat (FN_N_).  Table 3 shows the confusion matrix of the classification results.


(19) $$\begin{array}{c} TP_{N}=Nn, \end{array}$$

(20) $$\begin{array}{c} FP_{N}=Sn+Vn+Fn+Qn, \end{array}$$

(21) $$\begin{array}{c} TN_{N}=Ss+Sv+Sf+Sq+Vs+Vv+Vf+Vq+Fs+Fv+Ff+Fq+Qs+Qv+Qf+Qq, \end{array}$$

(22) $$\begin{array}{c} FN_{N}=Ns+Nv+Nf+Nq. \end{array}$$

In this paper, sensitivity, specificity, positive predictive value, and accuracy are used as indicators of classifier performance. Sensitivity (Se), also known as recall rate, is the proportion of positive samples that are correctly judged to be positive. The higher the sensitivity, the greater the proportion of samples correctly predicted. Specificity (Sp) is the proportion of correctly judged negative samples to actually negative samples. The positive predictive value (+*p*) refers to the proportion of correctly judged positive samples to all the judged positive samples. Accuracy (Acc) is the ratio of the sum of true positives and true negatives to the total number of samples, reflecting the consistency between test results and actual results. The calculation formula of the above four evaluation metrics is shown in (23–26).

(23) $$\begin{array}{c} Se=\frac{TP}{\left(TP+FN\right)}, \end{array}$$

(24) $$\begin{array}{c} Sp=\frac{TN}{\left(TN+FP\right)}, \end{array}$$

(25) $$\begin{array}{c} +p=\frac{TP}{\left(TP+FP\right)}, \end{array}$$

(26) $$\begin{array}{c} Acc=\frac{\left(TP+TN\right)}{\left(TP+TN+FP+FN\right)}. \end{array}$$

## 5. Results and Analysis

In order to build a time-series network model that is most suitable for the task of heartbeat classification and more accurately distinguish the categories of arrhythmias, we conducted the following five groups of experiments. In this section, we first compare and analyze the performance of RNN, GRU, and LSTM in heartbeat classification (Section 5.1). Secondly, the network is changed to bidirectional, and the classification results of BiRNN, BiGRU, and BiLSTM are compared (Section 5.2). Thirdly, by comparing the effects of different heartbeat lengths on the classification performance of the BiLSTM model, the optimal heartbeat length was selected (Section 5.3). Then, tree regularization was used to optimize the BiLSTM model. By adding tree regularization, the generalization ability of BiLSTM is improved, and the classification accuracy is improved, compared with the traditional L1 and L2 regularization (Section 5.4). Then, the important features of the simulated decision tree are analyzed and verified by experiments (Section 5.5). Finally, the results are compared with other references (Section 5.6).

### 5.1. Analysis of Experimental Results of Different Time-Series Networks

In order to select the optimal time-series network model, Experiment 1 selected three network models, namely, RNN, GRU, and LSTM, for heartbeat classification. The experimental results show that the overall classification accuracy of the RNN model and GRU model is 98.98% and 98.97%, respectively. The overall classification accuracy of the LSTM model is 99.09%, which is better than that of the RNN model and GRU model. However, it cannot fully consider the rhythm information by using the one-way recurrent neural network for heartbeat classification.  Table 4 shows the classification results and performance of three one-way recurrent neural networks.

### 5.2. Analysis of Experimental Results of Different Bidirectional Time-Series Networks

The one-way recurrent neural network can only learn the heartbeat information before the current moment when performing heartbeat classification. Therefore, we improve the selected LSTM network to BiLSTM so that the network can consider both the previous heartbeat information and the future heartbeat information. And the BiRNN and BiGRU networks are used for comparison and verification. The experimental results show that the overall classification accuracy of the BiRNN model and BiGRU model is 99.13% and 98.92%, respectively. The overall classification accuracy of the BiLSTM model is 99.18%, which is better than that of the BiRNN model and BiGRU model.  Table 5 shows the classification results and performance of the three bidirectional recurrent neural networks.

### 5.3. Select the Optimal Length of Heartbeat Segment

In order to select the optimal length of the heartbeat segment, a total of 7 experiments were conducted. The length of heartbeat segments selected by us is 1, 5, 10, 15, 20, 25, and 30, respectively, and the corresponding timestep of the BiLSTM is also 1, 5, 10, 15, 20, 25, and 30, respectively. The experimental results show that the classification accuracy of the network is gradually improved when the length of the heartbeat segment is less than 15. However, when the length of the heartbeat is greater than 15, the classification performance of the network decreases rapidly. The main reason is that the rhythm information of heartbeat, such as bigeminy, trigeminy, atrial tachycardia, and ventricular tachycardia, can be shown within 15 beats. When the heartbeat segment is too long, the heartbeat information considered by the network is too redundant, which will affect the network performance.  Table 6 shows the classification results of the BiLSTM network with different lengths of heartbeat segments.

### 5.4. Analyze the Experimental Results of Different Regularization Methods

In order to improve the generalization ability of BiLSTM and further improve the classification accuracy, we choose tree regularization to constrain the weight of the network and use the traditional L1 and L2 regularization for comparison. Experimental results verify the feasibility and effectiveness of the proposed model, and the overall classification accuracy is 99.32%. The overall classification accuracy of the models using L1 regularization and L2 regularization was 99.26% and 99.23%. Compared with Experiment 2, the overall accuracy of Experiment 4 was improved by 0.14%, and the precision of class S, class V, and class F was all improved, among which the precision of class F was improved more obviously by 5.62%. Through the above analysis, it is concluded that tree regularization can effectively improve the classification accuracy of the network, which is better than the traditional L1 and L2 regularization.  Table 7 shows the classification results of BiLSTM models under different regularization methods.  Figure 7 shows the confusion matrix of heartbeat classification results based on the BiLSTM-Treg model.

### 5.5. Analyze the Key Nodes of the Simulated Decision Tree

The tree regularization method used in this paper looks for the decision tree representation of the model in the training process of the network. The generated decision tree simulates the decision process of the BiLSTM network model. We call this decision tree a simulated decision tree (SDT). Since there are many feature points in a single heartbeat, the generated SDT is too large, so we selected the tree generated by the top 10 important feature points of SDT when displaying this decision tree, as shown in Figure 8. The top 10 important feature points are 126, 112, 162, 121, 153, 80, 224, 93, 100, and 120. The positions of these feature points corresponding to the ECG waveform are as follows: sampling points 126, 120, 121, and 153 correspond to ST segment, sampling point 112 to *J* point, sampling point 224 corresponds to the endpoint of *T* wave, sampling point 162 corresponds to the beginning point of *T* wave, sampling point 80 corresponds to the peak value of *Q* wave, sampling point 93 corresponds to the peak value of *R* wave, and sampling point 100 corresponds to the peak value of S wave, as shown in Figure 9.

In Figure 8, we have modified the representation of the value field in the decision tree node. We represent the value in the value field as the percentage of the number of heartbeats of N, S, V, F, and *Q* in the total number of heartbeats of the corresponding category. Taking node 2 as an example, 0.08 in the value field represents that the number of class S heartbeats in this node accounts for 0.08% of the total number of class S heartbeats, which means that this node almost contains no class S heartbeats. Therefore, according to this simulated decision tree, we have the following analysis:

1. Sampling point 126 is the root node of the simulated decision tree. According to whether the voltage value at this point is less than −0.0692 mV, the sample can be divided into two parts, namely, node 2 and node 3. In node 2, the heartbeat of classes F and *Q* is relatively large, while the heartbeat of the other three categories is relatively small. Therefore, 28.95% of class F heartbeats and 46.22% of class *Q* heartbeats were separated from the total sample according to the sampling point 126. Analysis of the reason: sampling point 126 is the point of ST segment in the ECG waveform. ST segment refers to the segment between the end of the QRS complex and the beginning of the *T* wave, representing the period between ventricular depolarization and ventricular repolarization [39]. The normal ST segment is smooth and flush with the baseline.
2. It is shown by nodes 11 and 12 that node 2 distinguishes the F heartbeats from the *Q* heartbeats according to the value of sampling point 224. There is only 0.38% of class *Q* heartbeat in node 11 and 0% of class S heartbeat in node 12. Analysis of the reason: sampling point 224 is the endpoint of *T* wave in the ECG waveform. *T* wave is a wave with a larger amplitude and longer duration after the QRS complex, which shows the process of ventricular repolarization.
3. It can be shown from node 5 that node 3 separates 25.1% of class V heartbeats and 25.53% of class *Q* heartbeats from node 3 according to the value of sampling point 112, and it is shown by node 14 and node 15 that node 5 distinguishes the heartbeats of class S from class *Q* according to the value of sampling point 153. Analysis of the reason: sampling point 112 is the *J* point in the ECG waveform, and *J* point is the junction point between the end of the QRS complex and the beginning of the ST segment.
4. As indicated by node 13, node 4 separates 26.00% of class V heartbeats from node 4 according to the value of sampling point 162. As indicated by node 16, node 6 separates 14.85% of class V heartbeats and 12.59% of class F heartbeats from node 6 according to the value of sampling point 80. Sampling point 162 and sampling point 80 are *T* wave start points and *Q* wave peak values, respectively.
5. It is shown by node 8 that 11.88% of N, 34.33% of S, 13.11% of V, 3.22% of F, and 19.53% of *Q* heartbeats are separated from the sample of node 7 according to the value of sampling point 93. After passing through nodes 9 and 10, 6.81% of class V is sorted out at node 18, 15.78% of class *Q* is sorted out at node 19, and 21.62% of class S heartbeat is sorted out at node 20. The reason is analyzed as follows: sampling point 93 and sampling point 100 are, respectively, *R* wave and S wave in ECG waveform, which together with *Q* wave corresponding to sampling point 80 constitute QRS complex. The QRS complex is a group of wave groups with complex changes and large amplitude, showing the process of ventricular depolarization [40].

To verify that the BiLSTM-Treg algorithm focuses on and learns from these medically significant feature points, in Experiment 5, we only used these 10 important feature points as the features of a single heartbeat and used the BiLSTM-Treg algorithm to classify the heartbeat. The experimental results are shown in Table 8, and the overall classification accuracy is 98.45%. Compared with Experiment 4, Experiment 5 showed no significant decrease in all other metrics except the sensitivity of class S. The experimental results validate the importance of these medically significant feature points in the model.

### 5.6. Comparison with Previous Studies

Table 9 compares the classification performance of this method and other literature methods. The experimental data of other pieces of literature also comes from the MIT-BIH arrhythmia database. It can be seen from Table 9 that the method proposed in this paper has the best classification accuracy, with an overall classification accuracy of 99.32%. The classification methods in literature [23, 25] all use the BiLSTM model. The results show that the proposed method has obvious advantages in all metrics except for the low sensitivity of class F, and the classification accuracy is 2.03% and 0.74% higher than the two methods, respectively. From the perspective of heartbeat type, the sensitivity of class S is significantly improved by the method presented in this paper compared with other methods. Compared with the literature [21], the method presented in this paper makes all metrics of *Q* heartbeat better, especially the sensitivity of *Q* heartbeat increased by 2.25%. In this paper, a classification method is proposed to integrate the rhythmic information between heartbeats that doctors are concerned about into the time-series network so that the network can learn this information effectively. Moreover, the bidirectional time-series network model can more conveniently obtain the context information of the heartbeat segment, so the algorithm in this paper can have better classification performance in the heartbeat classification problem.

## 6. Conclusion

In this paper, an intelligent classification of heartbeat based on the BiLSTM-Treg algorithm is proposed, which integrates rhythm information between heartbeats. This method fully considers the information of heart rhythm, which doctors pay attention to when diagnosing heart disease, and realizes the automatic classification of heartbeats. In this paper, the influence of different lengths of heartbeat segments on the classification results of the model is analyzed to select the best heartbeat segment length. On this basis, the BiLSTM-Treg algorithm was used for heartbeat classification. Experiments were carried out on the MIT-BIH arrhythmia database, and the results showed that the method can effectively distinguish five types of heartbeats, N, S, V, F, and *Q*, and the overall classification accuracy rate is 99.32%. The significance of this study is to provide patients with more accurate medical care services. The highlight of this study are as follows:

1. The heartbeat segment containing rhythm information between heartbeats was selected as the characteristics of the heartbeat sample, and the BiLSTM-Treg algorithm was used to automatically learn the potential rhythm information of individuals
2. A tree regularization method is proposed to optimize the BiLSTM-Treg algorithm and improve the accuracy of heartbeat classification
3. By analyzing the key nodes of the simulated decision tree, the interpretability of the BiLSTM-Treg algorithm is analyzed
4. The experimental results show that the algorithm proposed in this paper can effectively realize the classification of arrhythmia

In the future study, we will collect more class F-type heartbeat data for pretraining of the model so as to obtain more accurate intelligent ECG diagnosis results.

## Figures and Tables

**Figure 1:** The original ECG signal.

**Figure 2:** The denoised ECG signal.

**Figure 3:** Morphology of a single heartbeat and heartbeat segmentation.

**Figure 4:** The ECG signal with ventricular trigeminy.

**Figure 5:** The LSTM cell structure.

**Figure 6:** The BiLSTM model based on tree regularization.

**Figure 7:** Confusion matrix of heartbeat classification results based on the BiLSTM-Treg model.

**Figure 8:** The simulated decision tree.

**Figure 9:** The key feature points of the decision tree correspond to the positions in the ECG waveform.

**Algorithm 1:** The description of the BiLSTM-Treg model algorithm. BiLSTM-Treg model algorithm.

**Table 1:** Correspondence between MIT-BIH arrhythmia database annotations and AAMI heartbeat types.

AAMI heartbeat category	MIT-BIH heartbeat types
*N*	Normal beat (N); left bundle branch block beat (L); right bundle branch block beat (R); nodal (junctional) escape beat (j); atrial escape beat (e)
*S*	Aberrated atrial premature beat (a); nodal (junctional) premature beat (J); atrial premature beat (A); premature or ectopic supraventricular beat (S)
*V*	Premature ventricular contraction (V); ventricular escape beat (E)
*F*	Fusion of ventricular and normal beat (F)
*Q*	Paced beat (/); unclassifiable beat (Q); fusion of paced and normal beat (f)

**Table 2:** Experimental data statistics.

	Training set	Testing set	Total
*N*	81,551	9,044	90,595
*S*	2,501	280	2,781
*V*	6,519	716	7,235
*F*	723	79	802
*Q*	7,242	799	8041

**Table 3:** Classification results of heartbeat statistics.

Reference labels	Predicted labels				
	*n*	*s*	*v*	*f*	*q*
N	Nn	Ns	Nv	Nf	Nq
S	Sn	Ss	Sv	Sf	Sq
V	Vn	Vs	Vv	Vf	Vq
F	Fn	Fs	Fv	Ff	Fq
Q	Qn	Qs	Qv	Qf	Qq

**Table 4:** Comparison of the classification results of RNN, GRU, and LSTM network models.

	RNN				GRU				LSTM			
	Se (%)	Sp (%)	+*p* (%)	Acc (%)	Se (%)	Sp (%)	+*p* (%)	Acc (%)	Se (%)	Sp (%)	+*p* (%)	Acc (%)
*N*	99.61	97.10	99.35	99.15	99.45	97.80	99.51	99.15	99.69	97.40	99.42	99.27
*S*	90.40	99.80	92.86	99.54	92.72	99.77	92.11	99.58	92.05	99.90	96.19	99.68
*V*	97.66	99.80	97.26	99.66	97.94	99.76	96.61	99.63	96.98	99.77	96.84	99.59
*F*	71.26	99.94	91.18	99.72	71.26	99.91	86.11	99.68	75.86	99.91	86.84	99.72
*Q*	99.43	99.94	99.32	99.90	99.77	99.90	98.88	99.89	99.55	99.97	99.66	99.94

**Table 5:** Comparison of the classification results of BiRNN, BiGRU, and BiLSTM network models.

	BiRNN				BiGRU				BiLSTM			
	Se (%)	Sp (%)	+*p* (%)	Acc (%)	Se (%)	Sp (%)	+*p* (%)	Acc (%)	Se (%)	Sp (%)	+*p* (%)	Acc (%)
*N*	99.65	97.65	99.47	99.29	99.62	97.05	99.34	99.15	99.64	98.15	99.59	99.37
*S*	90.40	99.81	93.17	99.55	89.07	99.82	93.40	99.52	92.72	99.83	93.96	99.63
*V*	98.21	99.83	97.68	99.73	97.12	99.80	97.25	99.63	98.63	99.76	96.64	99.68
*F*	74.71	99.93	89.04	99.73	67.82	99.90	84.29	99.64	70.11	99.93	88.41	99.69
*Q*	100.00	99.97	99.66	99.97	99.77	99.91	98.99	99.90	100.00	99.98	99.77	99.98

**Table 6:** Effects of heartbeat segments of different lengths on the classification results of BiLSTM model.

Time step	1	5	10	15	20	25	30
Overall accuracy (%)	99.04	99.02	99.12	**99.18**	98.55	82.52	84.53

**Table 7:** Classification results of BiLSTM models based on different regularization methods.

	BiLSTM + *L*1				BiLSTM + *L*2				BiLSTM + Treg			
	Se (%)	Sp (%)	+*p* (%)	Acc (%)	Se (%)	Sp (%)	+*p* (%)	Acc (%)	Se (%)	Sp (%)	+*p* (%)	Acc (%)
*N*	99.73	98.00	99.55	99.41	99.73	97.80	99.51	99.38	99.78	97.95	99.54	99.44
*S*	91.72	99.90	96.18	99.67	91.72	99.89	95.85	99.66	93.38	99.91	96.58	99.73
*V*	98.63	99.81	97.42	99.73	98.49	99.78	97.02	99.70	98.63	99.83	97.69	99.75
*F*	74.71	99.92	87.84	99.72	72.41	99.96	94.03	99.74	72.41	99.96	94.03	99.74
*Q*	100.00	99.98	99.77	99.98	100.00	99.98	99.77	99.98	100.00	99.98	99.77	99.98

**Table 8:** Classification results based on key feature points and BiLSTM-Treg algorithm.

	Se (%)	Sp (%)	+*p* (%)	Acc (%)
*N*	99.28	95.45	98.98	98.58
*S*	77.81	99.61	85.14	99.01
*V*	97.94	99.74	96.35	99.62
*F*	73.56	99.93	88.89	99.72
*Q*	99.89	99.97	99.66	99.96

**Table 9:** Comparison with other studies.

	Reference	Classifier	Performance (%)
Feature engineering	Yang et al., 2021 [9]	Random forest	Acc = 98.1 Se = 75.2 +*p* = 93.9
	Ji et al., 2021 [15]	Stacking-DWKNN	Acc = 99.01 Se_n_ = 99.65; Sp_n_ = 94.94; +*P*_n_ = 99.38 Se_s_ = 89.42; Sp_s_ = 99.85; +*P*_s_ = 94.90 Se_v_ = 97.21; Sp_v_ = 99.78; +*P*_v_ = 97.07 Se_f_ = 80.77; Sp_f_ = 99.94; +*P*_f_ = 88.73
	Zhu et al., 2018 [7]	SVM	Acc = 97.80 Se_n_ = 99.27; +*P*_n_ = 98.48 Se_s_ = 87.47; +*P*_s_ = 95.25 Se_v_ = 94.71; +*P*_v_ = 95.22 Se_f_ = 73.88; +*P*_f_ = 86.09
Deep learning	Pandey et al., 2017 [21]	9-layer CNN	Acc = 94.03 Se_n_ = 91.54; Sp_n_ = 96.71; +*P*_n_ = 87.43 Se_s_ = 90.59; Sp_s_ = 98.63; +*P*_s_ = 94.30 Se_v_ = 94.22; Sp_v_ = 98.84; +*P*_v_ = 95.30 Se_f_ = 96.06; Sp_f_ = 98.67; +*P*_f_ = **94.76** Se_q_ = 97.75; Sp_q_ = 99.69; +*P*_q_ = 98.73
	Ji et al., 2019 [20]	1D-CNN	Acc = 99.21 Se_n_ = 98.27; Sp_n_ = **99.39** Se_v_ = 97.54; Sp_v_ = 99.44 Se_f_ = **98.07**; Sp_f_ = 99.50
	Wu et al., 2020 [23]	CNN-BiLSTM	Acc = 97.29 Se_n_ = 98.57; Sp_n_ = 93.62; +*P*_n_ = 98.81 Se_s_ = 84.97; Sp_s_ = 99.13; +*P*_s_ = 82.80 Se_v_ = 94.90; Sp_v_ = 99.35; +*P*_v_ = 94.00 Se_f_ = 76.89; Sp_f_ = 99.77; +*P*_f_ = 80.45
	Pandey et al., 2021 [25]	BiLSTM	Acc = 98.58 Se_n_ = 99.54; +*P*_n_ = 99.44 Se_s_ = 92.00; +*P*_s_ = 91.02 Se_v_ = 95.81; +*P*_v_ = 96.80 Se_f_ = 80.55; +*P*_f_ = 85.22
	Proposed	BiLSTM-Treg	Acc = **99.32** Se_n_ = **99.78**; Sp_n_ = 97.95; +*P*_n_ = **99.54** Se_s_ = **93.38**; Sp_s_ = **99.91**; +*P*_s_ = **96.58** Se_v_ = **98.63**; Sp_v_ = **99.83**; +*P*_v_ = **97.69** Se_f_ = 72.41; Sp_f_ = **99.96**; +*P*_f_ = 94.03 Se_q_ = **100.00**; Sp_q_ = **99.98**; +*P*_q_ = **99.77**

Bold values represent the best experimental results which correspond to the evaluation criteria for one certain type.

## Data Availability

(1) All datasets used to support the findings of this study are included within the paper. (2) All datasets used to support the findings of this study were supplied by the publicly available MIT-BIH database from the Massachusetts Institute of Technology. The URL to access this data is https://archive.physionet.org/cgi-bin/atm/ATM. (3) The coding used to support the findings of this study has not been made available because the source code in this paper is part of a national project and is a trade secret, so the source code is not available.

## References

[1] Atienza F. A., Morgado E., Martinez L. F., Alberola A. G., Alvarez J. L. R. (2013). Detection of life-threatening arrhythmias using feature selection and support vector machines. *IEEE Transactions on Biomedical Engineering*.

[2] Sannino G., De Pietro G. (2018). A deep learning approach for ECG-based heartbeat classification for arrhythmia detection. *Future Generation Computer Systems*.

[3] Mason R. E., Likar I., Biern R. O., Ross R. S. (1967). Multiple-lead exercise electrocardiography. *Circulation*.

[4] Saadatnejad S., Oveisi M., Hashemi M. (2019). LSTM-based ECG classification for continuous monitoring on personal wearable devices. *IEEE journal of biomedical and health informatics*.

[5] Wang J.-S., Chiang W.-C., Hsu Y.-L., Yang Y.-T. C. (2013). ECG arrhythmia classification using a probabilistic neural network with a feature reduction method. *Neurocomputing*.

[6] Hannun A. Y., Rajpurkar P., Haghpanahi M. (2019). Cardiologist-level arrhythmia detection and classification in ambulatory electrocardiograms using a deep neural network. *Nature Medicine*.

[7] Zhu W., Chen X., Wang Y., Wang L. (2018). Arrhythmia recognition and classification using ECG morphology and segment feature analysis. *IEEE/ACM Transactions on Computational Biology and Bioinformatics*.

[8] Zaorálek L., Platoš J., Snášel V. (2018). Patient-adapted and inter-patient ECG classification using neural network and gradient boosting. *Neural Network World*.

[9] Yang P., Wang D., Zhao W.-B., Fu L.-H., Du J.-L., Su H. (2021). Ensemble of kernel extreme learning machine based random forest classifiers for automatic heartbeat classification. *Biomedical Signal Processing and Control*.

[10] Qin Q., Li J., Zhang L., Yue Y., Liu C. (2017). Combining low-dimensional wavelet features and support vector machine for arrhythmia beat classification. *Scientific Reports*.

[11] Kutlu Y., Kuntalp D. (2012). Feature extraction for ECG heartbeats using higher order statistics of WPD coefficients. *Computer Methods and Programs in Biomedicine*.

[12] Ebrahimzadeh A., Ahmadi M., Safarnejad M. (2016). Classification of ECG signals using hermite functions and MLP neural networks. *Journal of AI and Data Mining*.

[13] Barhatte A. S., Ghongade R., Thakare A. S. QRS complex detection and arrhythmia classification using SVM.

[14] Ayar M., Sabamoniri S. (2018). An ECG-based feature selection and heartbeat classification model using a hybrid heuristic algorithm. *Informatics in Medicine Unlocked*.

[15] Ji S., Li R., Shen S., Li B., Zhou B., Wang Z. (2021). Heartbeat classification based on multifeature combination and Stacking-DWKNN algorithm. *Journal of Healthcare Engineering*.

[16] Wu M., Lu Y., Yang W., Wong S. Y. (2020). A study on arrhythmia via ECG signal classification using the convolutional neural network. *Frontiers in Computational Neuroscience*.

[17] Ganguly B., Ghosal A., Das A., Das D., Chatterjee D., Rakshit D. (2020). Automated detection and classification of arrhythmia from ECG signals using feature-induced long short-term memory network. *IEEE Sensors Letters*.

[18] Oh S. L., Ng E. Y. K., Tan R. S., Acharya U. R. (2018). Automated diagnosis of arrhythmia using combination of CNN and LSTM techniques with variable length heart beats. *Computers in Biology and Medicine*.

[19] Hou B., Yang J., Wang P., Yan R. (2019). LSTM-based auto-encoder model for ECG arrhythmias classification. *IEEE Transactions on Instrumentation and Measurement*.

[20] Ji Y., Zhang S., Xiao W. (2019). Electrocardiogram classification based on faster regions with convolutional neural network. *Sensors*.

[21] Acharya U. R., Oh S. L., Hagiwara Y. (2017). A deep convolutional neural network model to classify heartbeats. *Computers in Biology and Medicine*.

[22] Ashfaq Khan M., Kim Y. (2021). Cardiac arrhythmia disease classification using LSTM deep learning approach. *Computers, Materials & Continua*.

[23] Wu J., Li F., Chen Z., Xiang X., Pu Y. (2020). Patient-specific ECG classification with integrated long short-term memory and convolutional neural networks. *IEICE - Transactions on Info and Systems*.

[24] Li R., Zhang X., Dai H., Zhou B., Wang Z. (2019). Interpretability analysis of heartbeat classification based on heartbeat activity’s global sequence features and BiLSTM-attention neural network. *IEEE Access*.

[25] Pandey S. K., Janghel R. R. (2021). Classification of electrocardiogram signal using an ensemble of deep learning models. *Data Technologies and Applications*.

[26] Yildirim Ö. (2018). A novel wavelet sequence based on deep bidirectional LSTM network model for ECG signal classification. *Computers in Biology and Medicine*.

[27] Sawant C., Patii H. T. Wavelet based ECG signal de-noising.

[28] Alyasseri Z. A. A., Khader A. T., Al Betar M. A., Awadallah M. A. (2017). Hybridizing *β*-hill climbing with wavelet transform for denoising ECG signals. *Information Sciences*.

[29] Yao G., Mao X., Li N. (2021). Interpretation of electrocardiogram heartbeat by CNN and GRU. *Computational and Mathematical Methods in Medicine*.

[30] Verma A., Cabrera S., Mayorga A., Nazeran H. A robust algorithm for derivation of heart rate variability spectra from ECG and PPG signals.

[31] Donoho D. L., Johnstone I. M. (1994). Ideal spatial adaptation by wavelet shrinkage. *Biometrika*.

[32] Li W., Li J. (2017). Local deep field for electrocardiogram beat classification. *IEEE Sensors Journal*.

[33] Bsoul A. A. R., Ji S. Y., Ward K., Najarian K. Detection of P, QRS, and T components of ECG using wavelet transformation.

[34] Hochreiter S., Bengio Y., Frasconi P., Schmidhuber J. (2001). Gradient flow in recurrent nets: the difficulty of learning long-term dependencies. *Gradient Flow in Recurrent Nets: The Difficulty of Learning LongTerm Dependencies*.

[35] Hochreiter S., Schmidhuber J. (1997). Long short-term memory. *Neural Computation*.

[36] Schuster M., Paliwal K. K. (1997). Bidirectional recurrent neural networks. *IEEE Transactions on Signal Processing*.

[37] Wu M., Hughes M., Parbhoo S., Zazzi M., Roth V., Doshi Velez F. Beyond sparsity: tree regularization of deep models for interpretability.

[38] Apandi Z. F. M., Ikeura R., Hayakawa S. Arrhythmia detection using MIT-BIH dataset: a review.

[39] Kaplan Berkaya S., Uysal A. K., Sora Gunal E., Ergin S., Gunal S., Gulmezoglu M. B. (2018). A survey on ECG analysis. *Biomedical Signal Processing and Control*.

[40] Elgendi M. (2013). Fast QRS detection with an optimized knowledge-based method: evaluation on 11 standard ECG databases. *PloS one*.

